The article "Microscopic Interface and Multiscale Failure Analysis of Proposed Molecular Chain Polymers Based on Aifantis Strain Gradient Theory" was retracted in 2023. Reasons: signs of a paper mill; suspected computer-generated content; unreliable results or conclusions; concerns about the data.

# Microscopic Interface and Multiscale Failure Analysis of Proposed Molecular Chain Polymers Based on Aifantis Strain Gradient Theory

**DOI:** 10.1155/2022/1153080

**Published:** 2022-05-18

**Authors:** Chengxiang Li, Shuhu Li, GuiJie Yu

**Affiliations:** ^1^Shandong Non-metallic Materials Institute, Jinan 250031, Shandong, China; ^2^China University of Petroleum, Qingdao 266400, Shandong, China

## Abstract

A study on the microscopic morphology of real-world polymer blends and its mechanism of change showed that the microscopic morphology of equiproportional mixtures gradually changed from a dense body structure to a network structure with the addition of the total polymer concentration up to 20%; the microscopic morphology of mixtures with different proportions was characterized by the most uniform network structure of equiproportional mixtures when the total polymer concentration was 20%. The polymer acts as a defoamer in the mixed system. In this paper, the relationship between the microscopic morphology of each mixture and the physicochemical behavior of the two polymer chains in the mixed system was investigated on the basis of the Aifantis strain gradient theory. Molecular polymer microscopic interface and multiscale failure analysis are proposed. It is shown that for the dihedral angle distribution of four consecutive coarse-grained particles, the peaks obtained from all atomic-scale simulation data are reproduced in the coarse-grained model simulations. The deviation is within 2.5% in most places, except for the local area where the deviation exceeds 5%. Therefore, we have achieved good results for large-scale failures.

## 1. Introduction

Theoretical analysis, experimental measurement, and simulation have become the three main methods of modern scientific research [1]. With the rapid development of computer technology in recent years, computer simulation has been developing rapidly in the field of polymer science, covering almost all fields of polymer physics and chemistry [2]. However, for polymer systems, due to the long chain structure of polymers, their physical properties are multiscale in both time and space scales [3]. Therefore, it is difficult to study polymer molecular chain motion and stacking, crystallization and phase separation behavior, morphological evolution, and polymer rheological properties during processing by a theoretical or experimental method directly from microscopic to mesoscopic to macroscopic and microscopic scales [4]. With the rapid development of computer science and technology and the establishment of computer simulation methods at micro-, meso-, and macroscopic scales, it is possible to study polymer systems at multiple scales and has become the focus and frontier of polymer physics research today [5].

For polymer systems, the long chain structure of polymers makes their physical properties multiscale in both time and space scales [6]. The multiscale of polymers includes the spatial scale, i.e., from single molecule to the final molded material, such as the single bond length of the main chain of polymer chain is of human order of magnitude, while the radius of gyration of a single chain can reach the spit order of magnitude, and the size of the characteristic microphase area formed by the microphase separation of polymer block copolymer is several hundred, which is difficult to be realized under the current computer conditions if we want to study the mechanism of its formation from the atomic-level [7, 8]. The relaxation time spectrum spans one or twenty orders of magnitude. The time scales for polymer crystallization and growth often exceed 1 second, and phase separation of blends has even longer time scales [9]. It is a prospective and challenging topic that spans multiple scales from single-molecule design to materials processing and is also a new intersection and growth point for polymer science, condensed matter physics, materials science, and computational mathematics, which has important scientific significance and application prospects [10].

In order to study the properties of macromolecules at various scales, relatively mature theoretical systems and simulation methods have been developed at different scales in the microscopic, mesoscopic, and macroscopic aspects: the main simulation methods at the microscopic scale include molecular dynamics (MD) methods, Monte carlo simulation methods, Brownian dynamics (BD) methods, and dissipative particle dynamics (DP) [11, 12]. However, neither theoretical, simulation-based nor experimental has so far been a more mature method to put different through [13, 14]. Based on the development of the existing theoretical and simulation methods, we can establish different scale computer simulation methods for a specific polymer model system in time and space scales by establishing fine-grained and coarse-grained models of computer simulation methods and combining the results of theoretical and experimental studies, especially using experiments to fill the gap between different scales due to the limitations of theory and simulation, to realize the transition from microscopic to mesoscopic to macroscopic [15, 16]. In this paper, we combine the results of theoretical and experimental studies, especially the use of experiments to fill the gap between different scales caused by theoretical and simulation limitations, to achieve the coarse granulation from microscopic to mesoscopic to macroscopic and the fine granulation from macroscopic to mesoscopic to microscopic through computer simulation studies and then study the mesoscopic and macroscopic properties of polymer chains, to achieve the interface, and then lay the theoretical foundation for the design of polymer materials, the selection of processing conditions, and the optimization of performance [17, 18].

This paper presents the results of our research on the microscopic morphology of two water-soluble polymers in different concentrations of the same ratio and in different ratios of the same concentration, as well as the possible physicochemical behavior of the two polymer chains in the blended system [19, 20].

## 2. Coarse-Grained Multiscale through Simulation Study of Polymer Condensation

### 2.1. Multiscale Simulation Study of Coarse-Grained Polymers

In this method, the molecular dynamics of polymer chains is simulated at the full atomic scale, and the coarse-grained force field is obtained by Boltzmann-inversion based on the statistical radial distribution function and other distribution functions, and then the molecular dynamics of coarse-grained particles is simulated.

The radial distribution function is obtained from atomic simulation *g*(*r*), using Boltzmann transform as follows:

(1) $$\begin{array}{c} f\left(r\right)=-k_{B}T\;\ln\;g\left(r\right). \end{array}$$

Although it is not a potential energy, it can usually be used directly to extrapolate *V*_0_(*r*) and then iterate back as follows:

(2) $$\begin{array}{c} V_{i+1}\left(r\right)=V_{i}\left(r\right)+k_{B}T\;\ln\frac{g_{i+1}\left(r\right)}{g_{i}\left(r\right)}. \end{array}$$

Here, *g*_*i*_(*r*) is the radial distribution function obtained from the *i*-th iteration of the coarse-grained simulation.

### 2.2. Coarse-Grained Simulations of Nonstructural Properties

Coarse-grained simulations based on other nonstructural properties within the DPD framework mainly include coarse-grained simulations based on mechanical properties and coarse-grained simulations where DPD interaction parameters are obtained by fitting experimentally measurable properties.

Voth et al. proposed an elastic membrane-dissipative particle dynamics (EM-DPD) model; the bulk modulus, membrane area, and density obtained from atomic-level simulations are used to construct DPD particles. After the derivation, the force of particle *i* acting on particle *j* can be expressed as

(3) $$\begin{array}{c} F_{ij}^{c}=-\frac{8\omega }{r_{ij,0}^{2}}\left(\frac{r_{ij}-r_{ij,0}}{r_{ij,0}}\right)\hat{r_{ij}},\;\omega =\frac{h\lambda A_{0}}{2N\langle N_{\text{cut}}\rangle }. \end{array}$$

Here, *h* is the thickness of the membrane, *A*_0_ is the initial area of the membrane, *λ* is the bulk modulus of the membrane, and 〈*N*_cut_〉 is the average number of particles in the *r*_cutoff_ range of particle *i*. The remaining two required in the simulation *F*_*ij*_^*D*^ and *F*_*ij*_^*R*^ are of the same form as the forces required for the general simulation of DPD. Goot et al. called the interaction parameters required for the DPD simulation by fitting the experimentally measurable properties of compression coefficients, solubility parameters, and so on, so as to achieve the purpose of the DPD model to simulate the real material system. Firstly, from the water molecule *N*_*m*_ represented by each DPD particle, we obtained

(4) $$\begin{array}{c} r_{c}=3.107{\left(\rho N_{m}\right)}^{1/3}. \end{array}$$

By comparing with the experimental value of diffusion coefficient of water, the time unit of DPD was derived:

(5) $$\begin{array}{c} T=\left(14.1\pm 0.1\right)N_{m}^{5/3}. \end{array}$$

According to the formula,

(6) $$\begin{array}{c} \frac{1}{k_{B}T}{\left(\frac{\partial P}{\partial \rho }\right)}_{\mathrm{sim}.}=\frac{N_{m}}{k_{B}T}{\left(\frac{\partial P}{\partial n}\right)}_{\exp}. \end{array}$$

The interaction parameters between the same DPD particles can be derived:

(7) $$\begin{array}{c} a_{ij}=\frac{16N_{m}-1}{2\alpha \rho }. \end{array}$$

The interaction parameters *a*_*ij*_ between water and different macromolecules can be obtained from the experimental values of solubility parameters of water with a series of small hydrocarbon molecules, based on

(8) $$\begin{array}{c} \mu^{I}=\mu^{II}=\frac{\ln\left(\phi \right)}{N}-\ln\left(1-\phi \right)+\chi \left(1-2\phi \right),\\ p^{I}=p^{II}=\frac{\phi }{N}-\ln\left(1-\phi \right)-\phi -\chi \phi^{2}. \end{array}$$

The *X*-value for the interaction of water with this series of hydrocarbons was obtained to determine the value of Δ*a* and hence the value of *a*_*ij*_. Goot et al. performed simulations of cell membranes by this method, which is also applicable to real polymer systems for simulation.

## 3. Mesoscopic Simulation

In the coarse-grained model simulations of block copolymers, the efficiency of iterative fitting to different radial distribution functions decreases with increasing group size. Therefore, we also tried to perform multiscale simulations of block copolymers by combining molecular dynamics simulation methods and dissipative particle dynamics simulation methods. The simulations were carried out for a two-block copolymer of polystyrene-isoprene (*PS* − *b* − *PI*, (*SS*, *II* − *I*, *S* − *S* − *I*, *S* − *I* − *I*)) as an example.

### 3.1. Copolymer Model

When simulating the *PS* − *b* − *PI*-two-block copolymer, the most important thing is the selection of coarse-grained particles and the strategy of constructing the coarse-grained force field. In the next section, we describe in detail how the *PS* − *b* − *PI*-block copolymer model is constructed.

A basic assumption is that the volume of each DPD particle is equal. Therefore, specifically for the polystyrene-isoprene block copolymer, we first need to determine the monomer volumes of styrene and isoprene and then adopt an appropriate strategy to build the DPD particles. From the molecular volume calculation, we obtained the monomer volumes of styrene and isoprene as 159.4 Å^3^ and 135.3 Å^3^ and the volume of a water molecule at room temperature as 29.9 Å^3^, respectively. The monomer volumes of both styrene and isoprene are roughly equivalent to the volume of five water molecules. Therefore, in combination with the standard DPD particle coarse granulation strategy, we replaced one styrene monomer and one isoprene monomer with two different model DPD particles, as shown in Figure 1.

The time and space scales and temperature scales are expressed in the DPD simulations in terms of comparison units (reduced units) for simplicity; length units are expressed in terms of truncation radius *r*_*c*_ and energy units are expressed in terms of *k*_*B*_*T*. Here, the quantities represented in the simulation are estimated with respect to the real system. Since the real volume represented by a DPD simulation is approximately 150.0 Å^3^, the number density of DPD particles we use is equal to 3, which means that there are 3 DPD particles in a unit square, and the corresponding volume is approximately 450.0 Å^3^; the physical space scale of the particle interaction radius is $r_{c}=\sqrt[{3}]{450}=7.66\text{ Å}$.

Based on the work called by and, we estimate the time scale of

(9) $$\begin{array}{c} T=\left(14.1\pm 0.1\right)N_{m}^{5/3}=115.9\pm 0.1\text{ps}. \end{array}$$

In our simulation, the time step is Δ*t*=0.01_*T*_, so the time step of the simulation is equivalent to that in the real system.

Since mass, length, and energy are taken as comparative units, the temperature units can also be taken as comparative units. Thus, we can define *k*_*B*_*T*_0_=1.0, where *T*_0_ represents the room temperature. In this way, the interaction parameters in the simulation can be expressed in these comparative units. Then, we define another temperature to represent the comparison temperature.

### 3.2. Copolymer Coarse Graining Potential Field

In general, the force field used in molecular dynamics simulations of block copolymers at the all-atomic scale can be divided into two parts, the bonding part potential function and the nonbonding part potential function, and each part has different terms in terms of their contribution to the potential energy, as shown in equation (1). The coarse-grained force field required for the simulation of the block copolymer is constructed in a similar way, i.e., it consists of two major parts, namely, the bonding part interaction and the nonbonding part interaction. We use the bond length stretching energy and the bond angle bending energy to describe the bond part interaction; specifically, we take the form of the following simple resonance potential function:

(10) $$\begin{array}{c} F_{ij}^{S}=-k_{s}\left(r_{ij}-r_{s}\right){\hat{r}}_{ij},\\ F^{\theta }=-\nabla V_{\text{bend}},\\ V_{\text{bend}}=\frac{1}{2}k_{\theta }{\left(\theta -\theta_{0}\right)}^{2}, \end{array}$$

where *k*_*s*_ and *k*_*θ*_ denote the interaction coefficients of bond length and bond angle, respectively, and *r*_*s*_ and *θ*_*θ*_ denote the equilibrium distance of bond length interaction and the equilibrium bond angle of bond angle interaction, respectively. In addition, we use the conservative force term in to describe the nonbonded part interactions in the coarse-grained simulation system.

Bond part interaction parameters: we describe bond part interactions in terms of bond length stretching energy and bond angle bending energy. In order to establish the coarse-grained force field, first, we performed all-atom molecular dynamics simulations for the polystyrene-isoprene block copolymer. For the *PS* − *b* − *PI* block copolymer, we used two different types of DPD particles (*S*, *I* instead of styrene and isoprene monomers, respectively), which resulted in three different bond length distribution functions (*S* − *S*, *I* − *I*, *S* − *I*), four different bond angle distribution functions (*S* − *S* − *S*, *I* − *I* − *I*, *S* − *S* − *I*, *S* − *I* − *I*), and three different nonbonded part interaction distribution functions (*SS*, *II*, *SI*). For the distance distribution of two consecutive DPD particles, the bond length stretching energy can be obtained by Boltzmann transformation *V*_str_. The bond length part of the potential function is then discretized by smoothing to obtain the bond length part of the coarse-grained simulation. Similar to the bond length, for the bond angle distribution function of three consecutive DPD particles, we adjust the distribution function of this part by a weighting factor and then obtain the potential energy function of the bond angle part in the coarse-grained simulation by the Boltzmann transformation.

Based on these potential functions, we first simulated *PS* − *b* − *PI* and then counted the bond length distribution function and bond angle distribution function of the particles. We found that these distribution functions agree well with those obtained from all-atom molecular dynamics simulations, so we do not think it is necessary to carry out further optimization. The parameters of the bonding part action used in the simulations are shown in Table 1.

## 4. Considering Aifantis Strain Gradient Principal Structure Relationship

### 4.1. Classical Elastoplasticity Theory Intrinsic Structure Relationships

Commonly used large finite element simulation software such as ABAQUS and ANSYS have built-in intrinsic equations due to their macroscopic dimensions, and in addition, for all homogeneous linear elastic materials, the intrinsic relations can be expressed in matrix form as follows:

(11) $$\begin{array}{c} \sigma =C\varepsilon , \end{array}$$

where *σ*, *C*,  and *ε* are expressed in the matrix form as

(12) $$\begin{array}{c} \sigma^{T}=\left[\begin{array}{cccccc} \sigma_{x} & \sigma_{y} & \sigma_{z} & \tau_{xy} & \tau_{yz} & \tau_{zx} \end{array}\right],\\ \varepsilon^{T}=\left[\begin{array}{cccccc} \varepsilon_{x} & \varepsilon_{y} & \varepsilon_{z} & \gamma_{xy} & \gamma_{yz} & \gamma_{zx} \end{array}\right],\\ C=\frac{E\left(1-v\right)}{\left(1+v\right)\left(1-v\right)}\cdot \left[\begin{array}{c} 1,\frac{v}{1-v},\frac{v}{1-v},0,0,0\\ 1,\frac{v}{1-v},0,0,0\\ \frac{1-2v}{2\left(1-v\right)},0,0\\ \frac{1-2v}{2\left(1-v\right)},0\\ \frac{1-2v}{2\left(1-v\right)} \end{array}\right]. \end{array}$$

### 4.2. Aifantis' Strain Gradient Theory

The strain gradient term needs to be added to the macroscopic instanton equation since micro- and nanostructures already have significant size effects. Most of the strain gradient theories developed so far are second-order gradient theories, among which Aifantis' strain gradient theory is obtained by enhanced energy generalization, which can avoid the singularity of the strain domain and contains only one fine-scale material parameter, which is a simpler strain gradient theory with strong representativeness and stability and easy to apply. Aifantis used this theory to successfully explain the dimensional effects in deformation localization problems and torsion and bending problems [21, 22]. The intrinsic structure relationship after the introduction of strain gradient theory is

(13) $$\begin{array}{c} {\tilde{\sigma }}_{ij}=C_{ijkl}\left(\varepsilon_{kl}-l^{2}\nabla^{2}\varepsilon_{kl}\right). \end{array}$$

This section introduces the finite element implementation of the instanton equation with the introduction of strain gradient theory for a three-dimensional eight-node piezoelectric cell, so that the strain gradient instanton relationship for Aifantis can be expanded as

(14) $$\begin{array}{c} {\tilde{\sigma }}_{ij}=C_{ijkl}\varepsilon_{kl}-l^{2}C_{ijkl}\nabla^{2}\varepsilon_{kl}. \end{array}$$

Equation (14) can be further expanded as follows:

(15) $$\begin{array}{c} {\tilde{\sigma }}_{ij}=C_{ijkl}\varepsilon_{kl}-l^{2}C_{ijkl}\left(\frac{\partial^{2}\varepsilon_{kl}}{\partial x^{2}}+\frac{\partial^{2}\varepsilon_{kl}}{\partial y^{2}}+\frac{\partial^{2}\varepsilon_{kl}}{\partial z^{2}}+2\frac{\partial^{2}\varepsilon_{kl}}{\partial x\;\partial y}+2\frac{\partial^{2}\varepsilon_{kl}}{\partial y\;\partial z}+2\frac{\partial^{2}\varepsilon_{kl}}{\partial z\;\partial x}\right), \end{array}$$

where *C*_*ijkl*_ is the elastic constant of classical theory, *ε*_*kl*_ is the strain tensor component, and *l* is the inner Rin length coefficient.

Simplifying (15) into a matrix expression form and considering both thermal and electrical effects, the intrinsic relationship of the micropiezoelectric cell can be expressed as

(16) $$\begin{array}{c} \tilde{\sigma }=C\varepsilon -l^{2}C\left(\frac{\partial^{2}\varepsilon }{\partial x^{2}}+\frac{\partial^{2}\varepsilon }{\partial y^{2}}+\frac{\partial^{2}\varepsilon_{l}}{\partial z^{2}}+2\frac{\partial^{2}\varepsilon }{\partial x\;\partial y}+2\frac{\partial^{2}{}_{\varepsilon }}{\partial y\;\partial z}+2\frac{\partial^{2}{}_{\varepsilon }}{\partial z\;\partial x}\right)+A\cdot \Delta T+D\cdot E. \end{array}$$

For this three-dimensional eight-node cell, i.e., a hexahedral cell, using one Lagrangian polynomial and introducing three local coordinates *ξ*, *η*, *ζ* (−1 ≤ *ξ*, *η*, *ζ* ≤ 1), the form function of the three-dimensional eight-node cell can be constructed as

(17) $$\begin{array}{c} N_{i}=\frac{1}{8}1+\xi_{0}1+\eta_{0}\left(1+\zeta_{0}\right). \end{array}$$

Among them,

(18) $$\begin{array}{c} \xi_{0}=\xi_{i}\xi ,\\ \eta_{0}=\eta_{i}\eta ,\\ \zeta_{0}=\zeta_{i}\zeta . \end{array}$$

The partial derivative of the shape function with respect to the local coordinates can be expressed as

(19) $$\begin{array}{c} \frac{\partial N_{i}}{\partial \xi }=\frac{\partial N_{i}}{\partial x}\frac{\partial x}{\partial \xi }+\frac{\partial N_{i}}{\partial y}\frac{\partial y}{\partial \xi }+\frac{\partial N_{i}}{\partial z}\frac{\partial z}{\partial \xi }. \end{array}$$

For the other two local coordinates (*η*, *ζ*), the same expression can be obtained in the same way, written in matrix form as follows:

(20) $$\begin{array}{c} \left(\begin{array}{c} \frac{\partial N_{i}}{\partial \xi }\\ \frac{\partial N_{i}}{\partial \eta }\\ \frac{\partial N_{i}}{\partial \zeta } \end{array}\right)=\left(\begin{array}{ccc} \frac{\partial x}{\partial \xi } & \frac{\partial y}{\partial \xi } & \frac{\partial z}{\partial \xi }\\ \frac{\partial x}{\partial \eta } & \frac{\partial y}{\partial \eta } & \frac{\partial z}{\partial \eta }\\ \frac{\partial x}{\partial \zeta } & \frac{\partial y}{\partial \zeta } & \frac{\partial z}{\partial \zeta } \end{array}\right)\left(\begin{array}{c} \frac{\partial N_{i}}{\partial x}\\ \frac{\partial N_{i}}{\partial y}\\ \frac{\partial N_{i}}{\partial z} \end{array}\right)=J\left(\begin{array}{c} \frac{\partial N_{i}}{\partial x}\\ \frac{\partial N_{i}}{\partial y}\\ \frac{\partial N_{i}}{\partial z} \end{array}\right), \end{array}$$

where *J* is the Jacobi matrix, i.e., the partial derivative of the overall coordinates to the local coordinates.

In discretization of the general shape solution domain, the transformation relation between local and overall coordinates is

(21) $$\begin{array}{c} \begin{array}{c} x=\sum_{i=1}^{8}N_{i}x_{i},\\ y=\sum_{i=1}^{8}N_{i}y_{i},\\ z=\sum_{i=1}^{8}N_{i}z_{i}, \end{array}\;\left(i=1∼8\right), \end{array}$$

where *m* is the number of cell nodes where the coordinate transformation is performed.

*x*_*i*_, *y*_*i*_,  and *z*_*i*_ are the coordinate values of the nodes within the overall coordinates.

*N*_*i*_ is the form function expressed in local coordinates.

Using (21), *J* can also be expressed as a function of local coordinates as follows:

(22) $$\begin{array}{c} J=\left(\begin{array}{cccc} \frac{\partial N_{1}}{\partial \xi } & \frac{\partial N_{2}}{\partial \xi } & \ldots & \frac{\partial N_{8}}{\partial \xi }\\ \frac{\partial N_{1}}{\partial \eta } & \frac{\partial N_{2}}{\partial \eta } & \ldots & \frac{\partial N_{8}}{\partial \eta }\\ \frac{\partial N_{1}}{\partial \zeta } & \frac{\partial N_{2}}{\partial \zeta } & \ldots & \frac{\partial N_{8}}{\partial \zeta } \end{array}\right)\left(\begin{array}{ccc} x_{1} & y_{1} & z_{1}\\ x_{2} & y_{2} & z_{2}\\ \vdots & \vdots & \vdots \\ x_{8} & y_{8} & z_{8} \end{array}\right). \end{array}$$

Using the inverse matrix of the Jacobi matrix, the relationship between the overall coordinates of the form function pair and the local coordinates of the form function pair is as follows:

(23) $$\begin{array}{c} \left(\begin{array}{c} \frac{\partial N_{i}}{\partial x}\\ \frac{\partial N_{i}}{\partial y}\\ \frac{\partial N_{i}}{\partial z} \end{array}\right)=J^{-1}\left(\begin{array}{c} \frac{\partial N_{i}}{\partial \xi }\\ \frac{\partial N_{i}}{\partial \eta }\\ \frac{\partial N_{i}}{\partial \zeta } \end{array}\right),\;\left(i=1∼8\right). \end{array}$$

For a three-dimensional eight-node solid cell, each cell has 8 nodes, each node has 3 displacement components, and its cell node displacement array *a*^*e*^=[*u*_1_, *v*_1_.*w*_1_ … *u*_8_, *v*_8_, *w*_8_]^*T*^, such that

(24) $$\begin{array}{c} {\bar{N}}_{i}=\left(\begin{array}{ccc} N_{i} & 0 & 0\\ 0 & N_{i} & 0\\ 0 & 0 & N_{i} \end{array}\right),\;\left(i=1∼8\right). \end{array}$$

The above is the process of strain matrix construction based on strain gradient theory, and then performing the integration of the cell and overall cell matrix, the custom micropiezoelectric cell for the micro-piezoelectric captive is constructed [23, 24].

## 5. Experimental Analysis

### 5.1. Nonbonding Interaction

For the distance distribution of two consecutive coarse-grained particles, the bond length stretching energy V can be obtained by Boltzmann transformation, and then it is discretized by smoothing to obtain the bond length partial potential function in the coarse-grained simulation. Figures 2(a)–2(c) represent three different types of bond length distribution functions (*S* − *S*, *B* − *B*, *S* − *B*), respectively.

Similar to the bond length part, for the bond angle distribution function, we obtain the potential energy function of the bond angle part in the coarse-grained simulation by using a weighting factor sin(*α*) to rectify the distribution function of this part and then by Boltzmann transformation. Figures 3(a)–3(d) represent four different types of bond angle distribution functions (*S* − *S* − *S*, *B* − *B* − *B*, *S* − *S* − *B*, *S* − *B* − *B*), respectively.

This part is the most difficult to fit because the dihedral angle distribution is more influenced by the nonbonding interaction and the special nature of its own potential function. For the dihedral angle distribution of four consecutive coarse-grained particles, we still use the form of Fourier series to represent it. As can be seen from Figure 2, the peaks obtained from the all-atomic scale simulation data are reproduced in the coarse-grained model simulation. The deviations are within 2.5% in most places, except for local areas where the deviations exceed 5%. Therefore, we have obtained relatively good results for the dihedral angle fitting [25–27].

### 5.2. Potential Function for the Nonbonding Part

For this part, we refer to the extra potential to represent the nonbonding energy term and then use an iterative method to optimize the extra potential for the coarse-grained model. As can be seen in Figure 4, after several iterations, the radial distribution function obtained from the coarse-grained model simulation agrees well with the radial distribution function obtained from the all-atomic scale simulation.

We also analyzed the results of the full-atomic-scale simulations and coarse-grain model simulations of polystyrene butadiene from both static and dynamic aspects in the statistical process. We found that the relative errors of the mean square end distances and mean square radii of gyration obtained from the full-atomic-scale molecular dynamics simulations and the coarse-grained model simulations of polystyrene-butadiene block copolymers are within the range of the mean square end distances and mean square radii of gyration, which can indicate that our coarse-grained model is more effective.

The dynamics of polymer chains is also one of the core problems in polymer physics. In the simulation, we investigated the diffusion of one chain center of mass, which is a physical quantity describing the dynamics of polymer chains, and the diffusion curves obtained from the coarse-grained model simulation of polystyrene-butadiene block copolymer and the all-atomic scale simulation were in good agreement, which again verified the validity of our coarse-grained force field.

## 6. Conclusion

In this paper, we have described the relevant computational methods and their applications in establishing the coarse-grained force fields of block copolymers. The coarse-grained force field is obtained by performing molecular dynamics simulations of polymer chains at the full-atomic scale, and various distribution functions are calculated to establish a coarse-grained model. Finally, we statistically analyzed some physical quantities describing the properties of polymer chains, and the results proved the validity of the coarse-grained model. It is shown that the coarse granulation potential field can be used in the DPD mesoscopic simulations of polystyrene-isoprene two-block copolymers, where the styrene and isoprene monomers are coarse granulated into the same volume of DPD particles, respectively.

## Figures and Tables

**Figure 1:** Illustration of the CG apping of *PS* − *b* − *PI* diblock copolymer from atomistic to DPD model. s and I particles, respectively, represent the *PS* and *PI* block monomers.

**Figure 2:** Histograms of the (a) *S* − *S*, (b) *S* − *B*, and (c) *B* − *B* bond distributions of *PS* − *b* − *PB* obtained through atomistic (solid lines) and CG simulations (empty triangles).

**Figure 3:** Histograms of the (a) *S* − *S* − *S*, (b)*S* − *S* − *B*, (c)*S* − *B* − *B*, and (d)*B* − *B* − *B* angular distributions of *PS* − *b* − *PB* obtained through atomistic (solid lines) and CG simulations (empty squares).

**Figure 4:** Intrachain (a)*S* − *S*, (b)*S* − *B*, and (c)*B* − *B* radial distribution functions of *PS* − *b* − *PB* obtained through atomistic (solid lines) and coarse-grained simulations (empty squares), broken lines. (d) Optimized nonbonded numerical potentials obtained through coarse-grained simulations.

**Table 1:** The development of the interaction parameters from atomistic simulation to DPD scheme.

Interactions		AAMDsim.		DPDsim.	
Bonded terms	Bond length	*k*_*s*_(*k*_*B*_*T*)	*r*_0_(*nm*)	*k*_*s*_′(*n*_*w*_*k*_*B*_*T*/*R*_*C*_^2^)	*r*_0_′(*R*_*C*_)
	*S* − *S*	1.15	0.603	3.617	0.789
	*S* − *I*	22.07	0.588	72.001	0.658
	*I* − *I*	14.01	0.478	45.002	0.625
	Bond angle	*k*_*θ*_(1/rad^2^)	*θ*_0_(deg)	*k*_*θ*_′(*n*_*w*_*k*_*B*_*T*/rad^2^)	*θ*_0_′(rad)
	*S* − *S* − *S*	2.34	88.9	0.477	1.557
	*S* − *S* − *I*	11.22	71.09	0.628	1.251
	*S* − *I* − *I*	5.78	138.8	0.316	2.558
	*I* − *I* − *I*	1.32	125.5	0.075	2.188
Nonbonded terms	Repulsive force			*S*	*I*
	*S*			132.2	140.6
	*I*			141.3	132.5

## Data Availability

The raw data supporting the conclusions of this article will be made available by the authors, without undue reservation.
